# Targeting 3-Phosphoinoside-Dependent Kinase-1 to Inhibit Insulin-Like Growth Factor-I Induced AKT and p70 S6 Kinase Activation in Breast Cancer Cells

This article has been retracted.

**DOI:** 10.1371/journal.pone.0048402

**Published:** 2012-10-31

**Authors:** Sangita M. Baxi, Wei Tan, Sean T. Murphy, Tod Smeal, Min-Jean Yin

**Affiliations:** 1 Oncology Research, Pfizer Worldwide Research and Development, San Diego, California, United States of America; 2 Medicinal Chemistry, Pfizer Worldwide Research and Development, San Diego, California, United States of America; University of South Alabama, United States of America

## Abstract

Binding of IGF to IGF-IR activates PI3K to generate PIP3 which in turn recruits and activates proteins that contain a pleckstrin homology (PH) domain, including AKT and PDK1. PDK1 is highly expressed in breast tumor samples and breast cancer cell lines. Here we demonstrate that targeting PDK1 with the potent and selective PDK1 inhibitor PF-5177624 in the IGF-PI3K pathway blocks breast cancer cell proliferation and transformation. Breast cancer cell lines MCF7 and T47D, representing the luminal ER positive subtype and harboring *PIK3CA* mutations, were most responsive to IGF-I induction resulting in upregulated AKT and p70S6K phosphorylation via PDK1 activation. PF-5177624 downregulated AKT and p70S6K phosphorylation, blocked cell cycle progression, and decreased cell proliferation and transformation to block IGFR-I induced activation in breast cancer cells. These results may provide insight into clinical strategies for developing an IGFR-I inhibitor and/or a PDK1 inhibitor in luminal breast cancer patients.

## Introduction

The insulin-like growth factor (IGF) system is a complex set of interactions comprised of the ligands IGF-I and IGF-II, their corresponding receptors (IGFR-I and IGFR-II), IGF binding proteins 1–6 (IGFBPs), insulin receptor substrate (IRS), and related downstream pathways. The IGF signaling pathway plays a critical role in cellular proliferation and inhibition of apoptosis. Multiple studies using cultured breast cancer cells and xenograft or transgenic mouse models have demonstrated a critical role for IGF-IGFR signaling in breast cancer progression and metastasis [1], [2], [3], [4]. Many components of the IGF axis are altered in circulation and serve as important markers for prognosis and diagnosis in breast cancer patients [5], [6], [7]. In addition, activation of the IGF axis is implicated in the development of resistance to targeted therapies in breast cancer patients [8], [9], [10], [11]. Therefore, inhibition of IGF signaling pathways should be considered as potential targeted therapies for breast cancer treatment. Several small compound inhibitors and monoclonal antibodies targeting the IGF pathway have been investigated preclinically and/or are currently in early clinical development; these studies have provided evidence of anti-tumor activities in breast cancers [12], [13].

Binding of IGF to IGF-I receptor (IGF-IR) stimulates conformational change of the receptor and receptor tyrosine kinase activation, recruits and phosphorylates intracellular adaptor proteins such as IRS family members and SHC, and results in the activation of the PI3K pathway [12]. PI3Ks phosphorylate the D3 position of membrane phosphatidylinositides to generate phosphatidylinositol 3,4,5-triphosphate (PIP3); PIP3 serves as an important secondary messenger in the recruitment and activation of proteins that contain a pleckstrin homology (PH) domain, including AKT and 3′-phosphoinositide-dependent kinase-1 (PDK1). PDK1 is a 63-kDa Ser/Thr kinase with a catalytic domain near its N terminus and a pleckstrin homology domain at its C terminus. The pleckstrin homology domain is necessary for targeting PDK1 to the plasma membrane in order to phosphorylate the T-loop sites of numerous substrates, such as AKT at residue threonine-308 (T308). This T-loop activation at T308, along with phosphorylation of the serine-473 (S473) residue by mTORC2, fully activates AKT to induce downstream signaling pathways important for tumor progression [14], [15]. PDK1 has also been shown to phosphorylate p70S6K, isoforms of PKCs, and many other kinase substrates resulting in activation of downstream signaling and cell proliferation [14], [16].

The oncogenic activity of aberrant PI3K pathway signaling through PDK1 has been extensively studied. Hypomorphic mutation of PDK1 in PTEN+/− mice markedly protects these animals from developing a wide range of tumors [17]. Overexpression of PDK1 is sufficient to transform mammary epithelial cells [18] as well as potentiate ErbB2-induced transformation and migration [19], while down-regulation of PDK1 levels inhibits cell proliferation, survival, migration and metastasis of human breast cancer cells [20], [21]. In addition, knockdown of endogenous PDK1 in *PIK3CA* mutant breast cancer cells suppresses anchorage-independent growth, indicating a functional dependence on PDK1 in these cells [22]. Furthermore, PDK1 is highly expressed in a majority of human breast cancers and cell lines. Over 70% of invasive breast carcinomas express activated PDK1 at a moderate to high level [23], while 20% of breast tumors have five or more copies of the gene encoding PDK1 [19]. Additionally, elevated phosphorylation of PDK1 was associated with *PIK3CA* mutations in human breast tumor samples [22]. Consistent with the finding in tumor samples, PDK1 levels were also elevated in most breast cancer cell lines tested [19], [22]. Therefore, targeting PDK1 in the IGF-PI3K pathway may provide an additional opportunity for breast cancer treatment. In this study, we demonstrate that the selective and potent PDK1 inhibitor, PF-5177624, inhibits IGF-I stimulated AKT phosphorylation at residue T308 and the subsequent phosphorylation of downstream signaling molecules such as p70S6K. Inhibition of PDK1 activity is sufficient to induce anti-tumor activity in breast cancer cells such that PF-5177624 inhibits cell proliferation and cell transformation in these cells. Our data suggest that a selective and potent PDK1 inhibitor is likely to inhibit IGF-I driven tumorigenesis in breast cancer cells and moreover, that a PDK1 inhibitor should be evaluated as a therapeutic for breast cancer patients with elevated IGF-I activation.

**Figure 1:** IGF-I stimulated PDK1 activity in MCF7 and T47D cells. Breast cancer cell lines MCF7 and T47D were cultured in normal growth media (supplemented with 10% FBS) or serum starved for 24 hours. Growth factors EGF (**A**), TNFα (**B**)**,** IGF-I (**C**)**,** or insulin (**D**) were added to the culture media for 15 minutes after starvation. Cells were subsequently harvested and lysed, and lysates were subjected to SDS-PAGE. Western blot analysis was performed to examine the phosphorylation levels of AKT and p70S6K. GAPDH was included in each western blot analysis as a protein loading control.

## Materials and Methods

### PDK1 Inhibitors

PF-5177624 was synthesized as previously described [25]. PF-5177624 was dissolved in DMSO for all cellular assays.

**Figure 2:** PDK1 inhibitor PF-5177624 decreased IGF-I induced AKT and p70S6K phosphorylation. All IGF-1 stimulation experiments were subject to serum starvation for 24 hours prior to compound treatment or IGF-1 addition. MCF7 and T47D cells were stimulated with IGF-I at various time points, and phosphorylation levels of IGFR-I, AKT and p70S6K were determined (**A**). The structure of PF-5177624 is shown in **(B)**. MCF7 or T47D cells were pre-treated with the PDK1 inhibitor, PF-5177624 at 0.2 uM, 1 uM, or 5 uM for two hours prior to stimulation with IGF-I as noted. Cell lysates were prepared and subjected to SDS-PAGE. Western blot analysis were performed to determine the phosphorylation levels of IGFR-I, AKT, and p70S6K (**C**)**,** as well as PARP cleavage (**E**)**.** (**D**) Cells were cultured in a 96-well microtiter plate and treated with PF-5177624. After two hours of compound treatment, cells were stimulated with IGF-I (15 minutes) and cell lysates were analyzed by pAKT (T308) ELISA assay to determine the IC_50_ value of PF-5177624. The data shown for the cell treatments and western blots analysis are representative of at least two experiments.

### Cell Culture

BT20, HCC1954, MCF7, T47D, and MCF-10-2A cell lines were purchased from the American Type Culture Collection and cultured according to ATCC instructions. The gene mutation status of all cell lines was obtained from the Sanger COSMIC database: http://www.sanger.ac.uk/. Prior to stimulation, cells were cultured without serum for 24 hours. Cells were stimulated with EGF (100 ng/ml, Calbiochem/EMD Chemical), TNF-α, (50 ng/ml, R&D Systems), IGF-I (200 ng/ml, R&D Systems), or insulin (100 nM, Sigma-Aldrich) as indicated.

**Figure 3:** PF-5177624 blocked IGF-I induced cell cycle progression in MCF7 and T47D cells. Cells were serum-starved for 24 hours in order to synchronize cells at the G0/G1 stage. Cells were pre-treated with DMSO or PF-5177624 for 2 hours prior to addition of IGF-I for 6, 18, 24, 48, or 72 hours. Cells were subsequently harvested, fixed, and stained with PI and cell cycle profiles were obtained by flow cytometry. Bar graphs indicating the percentages of cells in the various cell cycle stages at the 72 hour time point are shown in (**A**) and (**B**)**.** Phosphorylation of Histone H3 was determined on cells treated with 5 µM PF5177624 for 24, 48, and 72 hours and normalized to DMSO treatment at the same time points as shown in (**C**). MCF7 and T47D cells were also incubated with BrdU and subject to FACS to measure incorporation of new DNA. The fold decrease of BrdU incoporation relative to DMSO treatment at the same time point are shown in (**D**). The t-test was performed to determine if there were differences in samples treated with compound versus DMSO at the same time point; *  =  p<0.05, **  =  p<0.001, ***  =  p<0.005.

**Figure 4:** PF-5177624 inhibited cell proliferation and cell transformation in MCF7 and T47D cells. Cells were cultured in complete medium and treated with PF-5177624 for 72 hours prior to addition of rezasurin to determine the IC_50_ value of cell proliferation inhibition by PF-5177624 (**A**)**.** Soft agar assays were performed in MCF7 (**B and C**) and T47D cells (**D and E**). The images from representative dishes and microscopy are shown to demonstrate colony numbers and morphology (**B and D**). Colony numbers were also counted (**C and E**).

### Immunoblotting

Cells were lysed in lysis buffer (150 mM NaCl, 1.5 mM MgCl_2_, 50 mM HEPES, 10% glycerol, 1 mM EGTA, 1% Triton X-100, 0.5% NP-40) supplemented with 1 mM Na_3_VO_4_, 1 mM PMSF, 1 mM NaF, 1 mM β-glycerophosphate, protease inhibitor cocktail (Roche), and phosphatase inhibitor cocktail (Roche) prior to use. Protein concentration was determined using the BCA Protein Assay (Pierce/Thermo Fisher Scientific) per the manufacturer’s instructions. Protein (30–50 µg) was resolved by SDS-PAGE and transferred onto nitrocellulose membrane. Blots were probed with primary antibodies to detect proteins of interest. After incubation with secondary antibodies, membranes were visualized by chemiluminescence (Pierce/Thermo Fisher Scientific). All antibodies were from Cell Signaling Technology, Inc with the exception of GAPDH (Santa Cruz Biotechnology) and phospho-p70S6K T252 (custom order). All western experiments were repeated at least two times.

### Cell Cycle Profiling

Cells were plated in six-well plates (100,000 cells/well) and allowed to adhere overnight prior to serum-starvation. After 24 hours of serum-starvation, compound was added for 2 hours and cells were then subjected to IGF-I stimulation for 6, 18, 24, 48, or 72 hours. At each time point, cells were collected, fixed, and permeablized using the Cell Cycle Phase Determination Kit (Cayman Chemical) following the manufacturer’s protocol. Samples were stored at −20°C until staining DNA with propidium iodide. Samples were also stained by anti-phosphorylated Histone H3 and anti-Bromodeoxyuridine (BrdU) to determine the number of cells in the mitotic and S phase stages. Anti-pH3 Fluor488-conjugated, anti-BrdU FITC-conjugated antibodies and BrdU were obtained from BD Bioscience and Sigma-Aldrich, respectively. Cells were labeled with 33 µM BrdU for 30 minutes before subjected to BrdU staining. A minimum of 10000 events were collected per sample on a BD FACSCalibur (BD Biosciences). Data analysis was done with FCS Express (De Novo Software). All assays were run in duplicate, and have been repeated at least twice.

### pAKT T308 ELISA

Cells were plated at 50,000 cells/well in a 96-well microtiter plate and allowed to adhere overnight. Cells were serum starved for 24 hours prior to compound treatment; PF-5177624 was added to each well (3-fold serial dilution starting at 10 µM) for two hours, followed by stimulation with IGF-I (15 minutes, 200 ng/ml) as noted. After compound treatment and stimulation, cells were lysed and lysate transferred to the ELISA plate. The pAKT T308 chemilumiscent ELISA was performed per the manufacturer’s directions (Cell Signaling Technology, Inc). All assays were run in duplicate, and have been repeated at least twice.

### Cell Proliferation

Cells were plated at 3,000 cells/well in a 96-well microtiter plate and allowed to adhere overnight. PF-5177624 was added to each well (3-fold serial dilution starting at 10 µM) and incubated for three days. At 72 hours post-compound addition, Resazurin (250 µg/ml final concentration, Sigma-Aldrich) was added to each well. Plates were incubated at 37°C for six hours and then analyzed for florescence (emission 590 nm, excitation 560 nm). All assays were run in duplicate, and have been repeated at least twice.

### Soft Agar Assay

MCF7 (50,000/well) and T47D (20,000/well) cells were plated for anchorage independent growth with compound in 0.35% BD Difco Noble agar (BD Diagnostic Systems) over a bottom layer of 0.5% BD Difco Noble agar containing MEM or RPMI, respectively. Cultures were maintained for a minimum of four weeks by weekly addition of compound in fresh agar (0.35%) containing medium. Microscope images of colony morphology were taken prior to colony visualization by addition of iodonitrotetrazolium chloride (1 mg/ml, Sigma-Aldrich) for 18 hours. Colonies were counted using the colony count function on the AlphaImager Gel Imaging System (Alpha Innotech/Protein Simple). All assays were run in duplicate, and have been repeated at least twice.

## Results

### IGF-I stimulates PDK1 Activity in Breast Cancer Cells

The mTORC2 complex directly phosphorylates AKT at S473 while PDK1 phosphorylates AKT at T308 [14], [24]. Therefore, pAKT-S473 is an indicator for PI3K/mTOR activity and pAKT-T308 is an indicator for PDK1 activity induced by RTKs. Similarly, specific phosphorylation sites in p70S6K correlate to the specific stimulatory activity of upstream kinases. Phosphorylation of p70S6K at T389 indicates activity stimulated by the mTORC1 complex, and phosphorylation at T252 indicates activation by PDK1 directly [14]. To investigate which RTK would stimulate the highest PDK1 activity, breast cancer cell lines HCC1954, BT20, MCF7, and T47D were treated with IGF-I, insulin, EGF or TNF-α, and phosphorylation levels of AKT and p70S6K were determined by western blot analysis (Figure 1 and Figure S1). All four tested breast cancer lines harbor *PIK3CA* mutations yet basal AKT phosphorylaton levels are not similar and induced AKT and p70S6K phosphorylation by RTKs are also different. The basal phosphorylation levels of both AKT and p70S6K are not significantly high in MCF7 and T47D cells, and are stimulated by EGF, IGF-I, and insulin but not by TNF-α. Among these four growth factors, IGF-I induced the highest activation of pAKT in MCF7 and T47D cells (Figure 1C). Furthermore, IGF-I was not able to induce phosphorylation of AKT and p70S6K in an untransformed mammary epithelial cell line, MCF-10-2A (Figure S1E). These results suggest that *PIK3CA* mutations in MCF7 and T47D cells do not lead to constitutive activation of downstream signaling but may enhance RTK stimulation signaling by activating high levels of phosphorylation of AKT and p70S6K in these cell lines. The highest phosphorylation levels of p70S6K at both T389 and T252 was observed primarily in MCF7 samples stimulated by EGF, IGF-I, and insulin. In T47D cells, however, phosphorylation of p70S6K upon IGF-1 stimulation is observed at T389 but not at T252. Taken together, these results suggest that PDK1 may play a critical role in IGF-I activated AKT and S6K phosphorylation in MCF7 and T47D cells.

### IGF-I induced Phosphorylation of AKT and p70S6K is Inhibited by a PDK1 Inhibitor

As previously reported, we have identified a potent and selective PDK1 inhibitor, PF-5177624 [25]. PF-5177624 has a K**_i_** value around 1 nM against PDK1 kinase activity in a biochemical assay and >100-fold selectivity against other PI3K/AKT pathway kinases. To further confirm our hypothesis that PDK1 plays a critical role in IGF-induced signaling in breast cancer cells, we used PF-5177624 (Figure 2B) to challenge the IGF-I induced signaling pathway. When MCF7 cells were treated with IGF-I, activation signals started at 15 minutes and were sustained up to 18 hours, but started to decline at 24 hours. Phosphorylation of IGFR at Y1135 increased ∼4–6 fold, AKT phosphorylation at both the S473 and T308 sites increased 8–12 fold, phosphorylation of p70S6K at T389 increased 2–3 fold, and phosphorylation of p70S6k at T252 increased around 2 fold (Figure 2A, Figure S2). In T47D cells treated with IGF-I, phosphorylation of IGFR at Y1135 increased 4–7 fold and AKT phosphorylation (S473 and T308) increased 3–6 fold, both for up to 24 hours. However, phosphorylation of p70S6K at T389 increased only 1.5–2 fold between 15 minutes and 2 hours and returned to basal levels after hour 6, while phosphorylation at T252 was not stimulated by IGF-I addition in T47D cells (Figure 2A, Figure S2).

Upon PF-5177624 pre-treatment for two hours, IGF-I induced pAKT (both S473 and T308) and pP70S6K (both T389 and T252) were markedly reduced in MCF7 (Figure 2C, Figure S2, and Table S1), and resulted in the increase of an apoptosis response as indicated by greater PARP cleavage in a dose-dependent manner at the three later time points (Figure 2E). The PDK1 inhibitor PF-5177624 did not inhibit the phosphorylation of IGFR in neither MCF7 nor T47D cells, indicating that the downregulation in phosphorylation of AKT and p70S6K is due to the specific inhibition of PDK1 (Figure 2C and Figure S2). PF-5177624 did inhibit IGF-I induced AKT phosphorylation at both the S473 and T308 sites in T47D cells, though inhibition was not observed at the 18 hour time point. Since phosphorylation of T252 in p70S6K was only minimally induced by IGF-I addition, PF-5177624 only inhibited pS6K at T389 in T47D cells (as shown in Figure 2C, Figure S2, and Table S2). Interestingly, although PF-5177624 inhibited pAKT (both S473 and T308) and pS6K (T389) in T47D cells, this inhibition did not induce PARP cleavage in T47D cells (Figure 2E). A quantitative ELISA to determine the phosphorylation of AKT at T308 was performed in IGF-I stimulated MCF7 and T47D cells and indicated that PF-5177624 dose-dependently inhibited pAKT at T308 with IC50 values of ∼400 nM and ∼700 nM in MCF7 and T47D, respectively (Figure 2D). PF-5177624 was also able to inhibit the phosphorylation of AKT and S6K in MCF7 and T47D cells grown under normal conditions (Figure S3). Therefore, a PDK1 inhibitor inhibited IGF-I induced activation of downstream signaling, including the phosphorylation of AKT and p70S6K, and resulted in the induction of PARP cleavage in MCF7 cells.

### A PDK1 Inhibitor Blocks IGF-I induced Cell Cycle Progression

Next, we looked at cell cycle progression to investigate whether the PDK1 inhibitor PF-5177624 was able to block IGF-I induced cell growth. MCF7 and T47D cells were serum starved for 24 hours to synchronize cells in the G0/G1 phase and then treated with PF-5177624 or DMSO two hours prior to IGF-I stimulation (200 ng/ml). Cells were harvested at the indicated time points post-stimulation and subjected to FACS analysis to determine cell cycle progression under IGF-I stimulation conditions. In MCF7 cells, IGF-I induced DNA synthesis with an increasing S phase starting at 18 hours and one cell cycle was completed at approximately 48 hours (Figure S4A). Addition of PF-5177624 in MCF7 cells decreased the cell population in the S phase and increased those in the G2/M block (Figure 3A and Table S3). In T47D cells, cell cycle progression induced by IGF-I started at 18 hours and lagged until 72 hours (Figure S4B); addition of PF-5177624 decreased the cell population in S phase and increased G0/G1 arrest (Figure 3B and Table S3). BrdU incorporation and phosphorylated Histone H3 staining assays were also performed to further confirm the decrease in S phase in MCF7 and T47D cells and G2/M block in MCF7 cells (Figure 3C and 3D). These results indicate that IGF-I stimulated different cell cycle progression profiles for MCF7 and T47D cells, and inhibition of PDK1 activity by PF-5177624 resulted in different patterns of cell cycle progression blockade whereby PF-5177624 leads to G2/M block in MCF7 cells and G0/G1 arrest in T47D cells. Furthermore, PF-5177624 also induced a subG1 cell population in both cell lines, suggesting that inhibition of PDK1 may induce cell apoptosis in both MCF7 and T47D cells (Figure 3, Figure 4 and Table S3). We have shown that PF-5177624 can induce PARP cleavage in MCF7 but not in T47D cells (Figure 2E), which suggests that it is likely that the apoptosis mechanism in T47D may be through an alternate mechanism other than PARP. The different cell cycle blockade patterns could be due to differences in downstream signaling inhibition by PF-5177624 in MCF7 and T47D cells, as we demonstrated that p70S6K phosphorylation at both T389 and T252 was stimulated by IGF-I and inhibited by PF-5177624 in MCF7 cells, but that there was not significant phosphorylation of p70S6K at T252 by IGF-I stimulation in T47D cells (Figure 2C).

### The PDK1 Inhibitor PF-5177624 Inhibits Cell Proliferation and Cell Transformation of Breast Cancer Cells

A cell proliferation assay was performed to determine whether PF-5177624 would demonstrate inhibition of cell growth under normal conditions (Figure 4A). IC_50_ values determined from the pAKT (T308) ELISA and cell proliferation assays treated with PF-5177624 are relatively similar, indicating a good correlation between kinase activity and cell proliferation. Furthermore, an anchorage independent growth assay was performed to evaluate whether inhibition of PDK1 activity would block cell transformation of MCF7 and T47D cells. Both MCF7 and T47D cells form colonies when cultured in soft agar, and addition of PF-5177624 decreased both colony size and colony numbers in the soft agar assay (Figure 4B–4E). The concentration needed to decrease colony formation was lower than the cell proliferation assay, and this observation is similar to previous reports in the literature where inhibition of PDK1 has a more profound effect on inhibition of cell transformation than cell proliferation [26]. We have demonstrated that PDK1 plays a critical role in the activation of AKT and p70S6K in MCF7 cells which may in part explain the better potency by PF-5177624 in inhibition of colony formation in MCF7 as compared to T47D cells.

## Discussion

PDK1 is downstream of PI3K and elevated phosphorylation of PDK1 has been associated with *PIK3CA* mutations in human breast tumor samples [22]. Therefore, we examined breast cancer cell lines with *PIK3CA* mutations in this study to investigate whether inhibition of PDK1 activity had antitumor effects in breast cancer cells subjected to growth factor stimulation. The breast cancer cell lines HCC1954 and BT20 are representative of triple negative breast cancer cells (TNBCs), while MCF7 and T47D cells represent luminal breast cancer cells. Although all four of these cell lines harbor a *PIK3CA* mutation, phosphorylation of AKT and p70S6K in MCF7 and T47D cells is not constitutively high and can be induced by IGF-I and other growth factors. These results highlight the difference in PI3K-AKT signaling in different breast cancer subtypes, and imply that growth factor stimulation may play an important role in luminal breast cancer cells harboring a *PIK3CA* mutation. Phosphorylation of AKT at T308 and p70S6K at T252 are indicators of PDK1 activity. Our data clearly show that IGF-I induced high levels of phosphorylation of AKT and p70S6K and that this activity could be modulated by inhibition of PDK1 activity in MCF7 cells. These data are also in line with recent publications demonstrating a role for IGF-IR/PDK1 signaling in the mediation of breast cancer cell growth [27], [28].

Cross-talk between the ErbB/HER family and the IGFR-I receptor signaling pathway has been described and suggested as a possible mechanism of resistance in breast cancer patients treated with the anti-HER2/neu antibody trastuzumab [10], [29]. IGFR-I signaling has also been implicated in the regulation of metastasis and invasion of breast cancer cells independent of tumor cell growth [2], [30]. However, IGFR-I upregulation of cell growth and cell cycle progression in ER positive breast cancer cells has not been well described with the exception of more recent publications [27], [31]. Results from our study further confirm that IGFR-I mediates cell proliferation through PDK1 activity in luminal breast cancer cells, and moreover, extend the evidence that the PI3K/AKT pathway is regulated by IGF-I stimulation in luminal but not triple negative breast cancer cells. This information is important and will assist development of clinical trial strategies in the design of combination therapies in different breast cancer subtypes.

Collectively, there are multiple pieces of evidence indicating that PDK1 plays an important role in mediating cell proliferation, transformation, migration and other oncogenic mechanisms as previously described. In this study, we further demonstrated that IGF-I induced cell proliferation is mediated by PDK1 activity in luminal breast cancer cells. Therefore, the driving mechanism of PDK1 mediated tumorigenesis may be cell type dependent or may be variable based on the genetic background of specific tumor cells. For example, a recent study used knockdown of PDK1 by an RNAi approach but did not observe a block in prostate or leukemia tumor development in PTEN-deficient transgenic mouse models [32]. As multiple kinases have been implicated as substrates of PDK1 [14], it is also likely that a PDK1 inhibitor, such as PF-5177624, would block IGF-I induced cell transformation by inhibiting multiple PDK1 substrates collaboratively in breast cancer cells. Moreover, another recent study suggests that direct interaction of PDK1 and IGFR-I in MCF7 cells may also provide insight into how a PDK1 inhibitor might block IGF-I induced signaling [27].

Several PDK1 inhibitors have been described [26], [33], [34]; however, these compounds lack cellular potency and reasonable kinase selectivity profiles. Here we demonstrate that a relatively potent and selective PDK1 inhibitor, PF-5177624, is able to inhibit IGF-I induced phosphorylation of downstream signaling molecules, block cell cycle progression, and decrease cell proliferation and transformation in luminal breast cancer cells. Although PF-5177624 does not have the desirable pharmacokinetic properties to perform animal studies, it serves as a good tool to investigate PDK1-mediated pathways. Further optimization of this series of PDK1 compounds is needed to conduct *in vivo* studies.

In conclusion, we have demonstrated that IGF-I signaling through the activation of PDK1 plays a critical role in the induction of cell cycle progression in luminal breast cancer cells. Furthermore, using the PDK1 inhibitor PF-5177624, we confirmed that inhibition of AKT and p70S6K can block IGF-I induced cell proliferation and transformation in MCF7 and T47D cells. These results provide evidence that inhibition of PDK1 may have greater anti-cancer therapeutic benefits in breast cancer patients with higher IGF-I/IGFR-I levels, and that a combination therapy featuring a PDK1 inhibitor and an IGFR-I inhibitor may have synergistic effects in this patient population.

## Supporting Information

Figure S1 Breast cancer cell lines HCC1954 and BT20 were cultured in normal growth media (with 10% FBS) or serum starved for 24 hours. Growth factors EGF **(A)**, TNFα **(B),** IGF-I **(C),** or insulin **(D)** were added to the culture media for 15 minutes after starvation. Cells were subsequently harvested and lysed, and lysates were subjected to SDS-PAGE. Western blot analysis was performed to examine the phosphorylation levels of AKT and p70S6K. An untransformed breast cell line, MCF-10-2A, was cultured in growth media with or without FBS and treated with IGF-I for 15 minutes after starvation. Cell lysates were evaluated by western blot to examine the phosphorylation levels of AKT and p70S6K **(E)**. GAPDH was included in each western as protein loading control.
(TIF)

Figure S2 The digital density of protein band in each western blot analysis was determined by FluorChem Q software for the blots shown in Figure 2A **(A)** and Figure 2C **(B)**. Relative activity of pIGFR, pAKT, and pS6K was determined by normalization of the density of the phosphorylated protein bands to GAPDH and total IGFR, AKT, and S6K. Data are from a representative experiment in MCF7 **(A)** and T47D **(B)**. Similarly, relative activity of pIGFR, pAKT, and pS6K after PF-5177624 treatments was calculated, and plotted by normalization to DMSO treated samples, and the graphs of 2 hour treatment were shown for MCF7 **(C)** and T47D **(D).** The t-test was performed to determine if there were any difference compared to the DMSO treatment group; *  =  p<0.05, **  =  p<0.001, ***  =  p<0.005.
(TIF)

Figure S3 MCF7 and T47D cells cultured in normal growth media were treated with 0.2, 1 or 5 µM of PF-5177624 at various time points, and phosphorylation levels of IGFR-I, AKT and p70S6K were determined by western blot.
(TIF)

Figure S4 Cells were serum-starved for 24 hours in order to synchronize cells at stage G0/G1. Cells were pre-treated with DMSO or PF-5177624 for 2 hours prior to addition of IGF-I for 6, 18, 24, 48, or 72 hours. Cells were subsequently harvested, fixed, and stained with PI and cell cycle profiles were obtained by flow cytometry. DNA content is shown in MCF7 **(A)** and T47D **(B)**.
(TIF)

Table S1 The detailed relative activity changes of pIGFR-I, pAKT and pS6K by PF-5177624 treatment in MCF7 cells at all time points are summarized.
(TIF)

Table S2 The detailed relative activity changes of pIGFR-I, pAKT and pS6K by PF-5177624 treatment in T47D cells at all time points are summarized.
(TIF)

Table S3 The detailed cell population at the various cell cycle stages at each time point are summarized in MCF7 and T47D cells.
(TIF)
